The article "Role of high expression levels of STK39 in the growth, migration and invasion of non-small cell type lung cancer cells" was retracted in 2026. Reasons: plagiarized images; duplicated images; overlap with other authors' work; original data or images not available.

# Role of high expression levels of STK39 in the growth, migration and invasion of non-small cell type lung cancer cells

**DOI:** 10.18632/oncotarget.11351

**Published:** 2016-08-17

**Authors:** Zhao Li, Wenzhuo Zhu, Liwen Xiong, Xiaobo Yu, Xi Chen, Qiang Lin

**Affiliations:** ^1^ Department of Thoracic Surgery, Shanghai General Hospital, Shanghai Jiaotong University School of Medicine, Shanghai, China; ^2^ Department of Pulmonary Diseases, Shanghai Chest Hospital, Shanghai Jiaotong University School of Medicine, Shanghai, China

**Keywords:** STK39, NSCLC, proliferation, metastasis

## Abstract

Non-small cell type lung cancer (NSCLC) is the most common malignancy and the leading cause of cancer related mortality. In this study, serine/threonine kinase 39 (STK39) was identified as an up-regulated gene in NSCLC tissues by next-generation RNA sequencing. Although STK39 gene polymorphisms may be prognostic of overall survival in patients with early stage NSCLC, the roles of STK39 in NSCLC cancer are poorly understood. In the current study, Genome Set Enrichment Analysis (GSEA) on the RNA-seq data of NSCLC specimens indicated that cancer-related process and pathways, including metastasis, cell cycle, apoptosis and p38 pathway, were significantly correlated with STK39 expression. STK39 expression was significantly increased in NSCLC cases and its protein expression was positively correlated with the poor tumor stage, large tumor size, advanced lymphnode metastasis and poor prognosis. Down-regulation of STK39 in NSCLC cells significantly decreased cell proliferation by blocking of cell cycle and inducing apoptosis. We also found that STK39 knockdown in NSCLC cells remarkably repressed cell migration and invasion. On the contrary, overexpression of STK39 in NSCLC cells had inverse effects on cell behaviors. Taken together, STK39 acts as a tumor oncogene in NSCLC and can be a potential biomarker of carcinogenesis.

## INTRODUCTION

Lung cancer is the most common malignancy and the leading cause of cancer related mortality both in China and worldwide [1, 2]. Histologically, more than 80% of lung cancers are non-small cell type lung cancer (NSCLC), which includes adenocarcinoma (ADC), squamous cell carcinoma (SCC), large cell carcinoma (LCC) and others [3]. In the last few decades, with the advances in our knowledge of the molecular biology of tumors, targeted therapy has become an important strategy for treating lung cancer. However, the prognosis of NSCLC patients with locally advanced or metastatic disease remained ominous [2]. Thus, identifying novel diagnostic and prognostic markers using a more comprehensive approach would facilitate the development of new strategies for new therapeutic targets for NSCLC treatment.

The article "Role of high expression levels of STK39 in the growth, migration and invasion of non-small cell type lung cancer cells" was retracted in 2026. Reasons: plagiarized images; duplicated images; overlap with other authors' work; original data or images not available.

Next-generation RNA sequencing (RNA-Seq) has become a powerful tool to identify biomarkers and understand tumorigenesis at the molecular level [4–6]. Here, we applied RNA-Seq to sequence the whole transcriptomes of 10 pairs of NSCLC and adjacent non-cancerous specimens. We identified serine/threonine kinase 39 (STK39), a member of the Ste20-like kinase family [7], as an up-regulated gene in NSCLC tissues as compared with non-cancerous tissues. STK39 appears to act as MAPK kinase kinase kinases (MAP4K) and was thought to be involved in stress response via activating p38 MAPK [8]. In patients with primary prostate cancers who received radical prostatectomy, the lower mRNA expression of STK39 was strongly associated with the higher incidence of metastases [9]. In early-stage NSCLC, two single-nucleotide polymorphisms (rs10176669 and rs4438452) located in STK39 gene may be prognostic of overall survival [10]. However, the roles of STK39 in NSCLC cancer remain unknown. Genome Set Enrichment Analysis (GSEA) on the RNA-seq data of NSCLC specimens indicated that STK39 expression was significantly correlated with cancer-related process and pathways, which suggest the involvement of STK39 in the progression of NSCLC. We then revealed the clinical values of STK39 in NSCLC. Further *in vitro* cell functional experiments and *in vivo* animal experiments suggested that STK39 might serve as an oncogene by increasing cell proliferation, migration and invasion.

## RESULTS

### RNA-seq analysis of 10 matched pairs of NSCLC and adjacent non-cancerous tissues

We performed RNA-seq on 10 pairs of NSCLC and adjacent non-cancerous lung tissues using the Illumina platform. Genes exhibiting greater than 1.5-fold differentially expressed with a *P* value less than 0.05 were defined as differential expressed genes (DEGs). Here, 7,220 DEGs were identified with 3,752 up-regulations (Supplementary Table S1) and 3,468 down-regulations (Supplementary Table S2) in NSCLC tissues, when compared with non-cancerous tissues (Figure 1A).

**Figure 1:** RNA sequencing data analysis (**A**) DEGs were identified by RNA sequencing. (**B**) RNA-sequencing data showed that STK39 mRNA expression was significantly higher in NSCLC tissues than in paired non-cancerous tissues (*n* = 10). (**C**) GSEA analysis in NSCLC patients with higher STK39 expression versus lower STK39 expression. NES, normalized enrichment score.

Among the DEGs, STK39, a member of the Ste20-like kinase family [7], was previously reported to be associated with the prognosis of early-stage NSCLC [10] (Figure 1B). GSEA on the RNA-seq data of NSCLC tissues indicated that cancer-related process and pathways (Supplementary Table S3 and Figure 1C), such as metastasis, cell cycle, apoptosis and p38 pathway, were significantly enriched in STK39 higher expression tissues. These data suggested that STK39 may be involved in the progression of NSCLC.

The article "Role of high expression levels of STK39 in the growth, migration and invasion of non-small cell type lung cancer cells" was retracted in 2026. Reasons: plagiarized images; duplicated images; overlap with other authors' work; original data or images not available.

### Up-regulated STK39 expression correlates with poor survival of patients with NSCLC

To investigate STK39 expression patterns in NSCLC, we first examined mRNA levels of STK39 in 40 pairs of NSCLC and adjacent non-cancerous tissues by using real-time PCR. The results showed that STK39 expression significantly higher in NSCLC tissues than in non-cancerous tissues (Figure 2A). Similar results were observed after re- analyzing gene expression data downloaded from The Cancer Genome Atlas website (TCGA, https://tcga-data.nci.nih.gov/tcga/, Figure 2B). Results of Western blot (Figure 2C) and immunohistochemistry (IHC, Figure 2D) analyses showed that STK39 was abundant in NSCLC tissues at protein level.

**Figure 2:** STK39 overexpression correlates with poor survival in patients with NSCLC (**A**) STK39 mRNA levels were determined in 40 pairs of NSCLC and non-cancerous tissues using real-time PCR. (**B**) STK39 expression in lung adenocarcinoma and normal tissues based on TCGA dataset (*P* < 0.0001). (**C**) Representative STK39 protein expression in unaffected tissues (N1, N2, N3 and N4) and NSCLC (T1, T2, T3 and T4). (**D**) STK39 protein expression was assessed by immunohistochemistry staining in NSCLC tissues. Scale bar: 100 μm. (**E**) Kaplan-Meier survival analysis showed that patients with lower STK39 expression level have a better prognosis than that of patients with higher STK39 expression (*P* < 0.01).

Further, according to IHC results, the 135 patients were categorized into two groups: lower expression group (less than 20% of tumor cells were positively stained, *n* = 58) and higher expression group (more than 20% of tumor cells were positively stained, *n* = 77). To explore the clinical significance of STK39 in NSCLC, we analyzed the correlation between STK39 expression levels and patients' features by using Fisher's exact test. The results indicated that STK39 expression was significantly correlated with tumor size (*P* = 0.0045), tumor stage (*P* = 0.0302) and lymph node metastasis (*P* = 0.0146). While, there is no correlation between STK39 expression level and age, gender or tumor type (Table 1).

**Table 1:** Correlation of STK39 protein expression with patients' features

Variables	All cases	STK39 protein		*P* value
		Low (*n* = 58)	High (*n* = 77)	
**Age at surgery**				
< 55	38	24	29	0.7231
> = 55	97	34	48	
**Gender**				
Male	72	30	42	0.8618
Female	63	28	35	
**Tumor size**				
< 3 cm	55	32	23	0.0045**
> = 3 cm	80	26	54	
**Tumor type**				
SCC	71	33	38	0.1707
ADC	46	15	31	
LCC	18	10	8	
**Tumor stage**				
I + II	85	43	42	0.0302*
III	50	15	35	
**Lymph node metastasis**				
Absent	74	39	35	0.0146*
Present	61	19	42	

Abbreviations: SCC, squamous cell carcinoma; ADC, adenocarcinoma; LCC, large cell carcinoma.

* *P* < 0.05,

** *P* < 0.01.

The article "Role of high expression levels of STK39 in the growth, migration and invasion of non-small cell type lung cancer cells" was retracted in 2026. Reasons: plagiarized images; duplicated images; overlap with other authors' work; original data or images not available.

We then investigated the correlation between STK19 protein expression and prognosis of NSCLC patients. Kaplan-Meier analysis showed that patients with lower STK39 expression had longer overall survival time than those with higher STK39 expression (Figure 2E).

### STK39 promotes the proliferation of NSCLC cells

To investigate the functional role of STK39 in NSCLC cells, firstly, the expression of STK39 in diverse NSCLC cell lines was detected. As illustrated in Figure 3A and 3B, NCI-H358 and NCI-H1975 cells exhibited higher expression of STK39 at both mRNA and protein levels, whereas A549 showed lower expression.

**Figure 3:** STK39 promotes cell proliferation in NSCLC cells (**A**, **B**) STK39 protein and mRNA expression in 5 NSCLC cell lines was analyzed by Western blot (A) and real-time PCR (B), respectively. Data were based on at least 3 independent experiments. (**C**) Expression of STK39 in NCI-H358, NCI-H1975 and A549 cells was analyzed by Western blot. NCI-H358 and NCI-H1975 cells were transfected with STK39 siRNA (siRNA3) or control siRNA (siNC); A549 cells was infected with STK39 expression lentivirus or control vector lentivirus (Vector). (**D**) Cell proliferation was detected at 0, 24, 48 and 72 h after siRNA transfection or lentiviral infection in NCI-H358, NCI-H1975 and A549 cells. Data were based on at least 3 independent experiments, and shown as mean ± SD. ***P < 0.001.

Next, we knocked down endogenous STK39 expression by siRNA transfection in NCI-H358 and NCI-H1975 cells, but overexpressed STK39 in A549 cells (Supplementary Figure S1 and Figure 3C). CCK-8 assay was performed to measure the capability of cell proliferation. Knockdown of STK39 in NCI-H358 and NCI-H1975 cells caused a significant decrease in the cell proliferation at 48 and 72 h after siRNA transfection. While, overexpression of STK39 in A549 cells by lentiviral infection significantly increased cell proliferation rate (Figure 3D). These data indicated that STK39 was able to promote the proliferation of NSCLC cells.

### STK39 promotes G1/S cell cycle transition and decreases the apoptosis of NSCLC cells

As described above, GSEA results showed that cell cycle and apoptosis pathway were strongly associated with STK39-higher expression (Figure 1C). Thus, we explored the effects of STK39 on cell cycle and apoptosis of NSCLC cells. Cell cycle profile analysis revealed that STK39 siRNA transfection in NCI-H358 and NCI-H1975 cells led to a significant increase in the population of G0/G1 phase and a remarkably decrease in the percentages of S and G2/M phase cells. While, STK39 overexpression in A549 cells significantly decreased the percentages of cells in G0/G1 phase (Figure 4A).

The article "Role of high expression levels of STK39 in the growth, migration and invasion of non-small cell type lung cancer cells" was retracted in 2026. Reasons: plagiarized images; duplicated images; overlap with other authors' work; original data or images not available.

**Figure 4:** STK39 accelerates G1/S phase transition and inhibits cell apoptosis in NSCLC cells NCI-H358 and NCI-H1975 cells were transfected with STK39 siRNA (siRNA3) or control siRNA (siNC); A549 cells was infected with STK39 expression lentivirus or control vector lentivirus (Vector). At 24 h after siRNA transfection or lentiviral infection, cells were collected. (**A**) Cell cycle distribution was analyzed using PI staining and flow cytometry. (**B**) Cell apoptosis was measured by Annexin V-PI double staining followed by flow cytometry analysis. **P < 0.01, ***P < 0.001.

The inactivation of STK39 has also been shown to enhance cell to apoptosis [11, 12]. Annexin V-FITC/PI staining assay revealed that knockdown of STK39 in NCI-H358 and NCI-H1975 cells significantly induced cell apoptosis. While, overexpression of STK39 had the opposite effect on the apoptosis of A549 cells (Figure 4B). These results indicated that STK39 may promote NSCLC cell proliferation by stimulating G1/S cell cycle transition and impeding cell apoptosis.

### STK39 promotes the migration and invasion of NSCLC cells

The migration and invasion capacity was then evaluated by Transwell assay with non-Matrigel-coated and Matrigel coated Transwell inserts, respectively. As shown in Figure 5, transfection of STK39 siRNA3 into NCI-H358 and NCI-H1975 cells significantly reduced the migration and invasion ability compared with siNC. On the contrary, STK39 overexpression in A549 cells promoted cell migration and invasion.

**Figure 5:** STK39 promotes the cellular migration and invasion of NSCLC cells Migration (**A**) and invasion (**B**) assay were performed in Transwell chambers. For invasion assay, the upper chamber was pre-coated with Matrigel. Scale bar: 100 μm ***P < 0.001.

### STK39-associated pathways in NSCLC

As mentioned above, GSEA results showed that cancer-related process and pathways were significantly enriched in STK39 higher expression tissues (Supplementary Table S3 and Figure 1C). To further validate the GSEA results, we then detected the protein expression of cell cycle (PCNA and CDC25A), cell apoptosis (Bcl-2 and Bax) and metastasis (MMP-2, MMP-9, Snail and E-cadherin) in NSCLC cells (Figure 6A). The expression of PCNA, CDC25A, Bcl-2, MMP-2, MMP-9 and Snail was significantly decreased, while Bax and E-cadherin expression was notably increased in both NCI-358 and NCI-H1975 cells after STK39 knockdown. The reversed effects were observed in A549 cells infected with STK39 expressing virus.

The article "Role of high expression levels of STK39 in the growth, migration and invasion of non-small cell type lung cancer cells" was retracted in 2026. Reasons: plagiarized images; duplicated images; overlap with other authors' work; original data or images not available.

**Figure 6:** Mechanisms how STK39 exerts its function in NSCLC NCI-H358 and NCI-H1975 cells were transfected with STK39 siRNA (siRNA3) or control siRNA (siNC); A549 cells was infected with STK39 expression lentivirus or control vector lentivirus (Vector). (**A**) At 48 h after siRNA transfection or lentiviral infection, cells were collected. Protein levels of key proteins in cell cycle, cell apoptosis and metastasis were determined by Western blot. Representative blots of 3 independent experiments were shown. (**B**) Phosphorylation of p38 was detected by Western blot.

STK39 appears to activate MAPK/p38 [8], which is selectively activated in human NSCLC tissues [13]. We then examine the effect of STK39 on p38 phosphorylation. In NCI-358 and NCI-H1975 cells transfected with STK39 siRNA3, p38 phosphorylation was significantly reduced as compared to cells transfected with siNC. Inversely, over-expression of STK39 in A549 cells dramatically increased the phosphorylation status of p38 (Figure 6B).

### STK39 knockdown suppresses tumorigenesis of NSCLC cells in nude mice xenograft model

Next, we determined whether knockdown of STK39 in NSCLC cells could reduce tumor growth *in vivo*. NCI-H358 cells stably infected with STK39 knockdown lentivirus (shSTK39) or control lentivirus (shNC) were subcutaneously injected into nude mice. As shown in Figure 7A and 7B, STK39 silenced tumors grew much slower and the size was much smaller than control tumors at 27 days after cell inoculation. Further, a significant decrease of Ki67-positive cells and a notable increase of apoptotic cells were observed in STK39 silenced tumors, as compared to control tumors (Figure 7C). These data suggested that knockdown of STK39 inhibited tumor growth in nude mice.

**Figure 7:** STK39 knockdown suppressed NSCLC cell proliferation *in vivo* Knockdown of STK39 in NCI-H358 cells significantly inhibited tumor growth in nude mice xenograft model. (**A**) The growth curves of xenograft tumors in different groups. (**B**) At day 27, mice were sacrificed and tumors were resected (*n* = 6). Comparison of excised tumors. Scale bar: 1 cm. (**C**) Xenograft tumors with Ki67 immunostaining and TUNEL staining. Scale bar: 100 μm. *P < 0.05, **P < 0.01, ***P < 0.001.

## DISCUSSION

In this study, we conducted RNA sequencing for 10 pairs of NSCLC and non-cancerous lung tissues, and identified a novel DEG, STK39. GSEA revealed that STK39 expression in NSCLC tissues was strongly associated with cancer-related process and pathways (Figure 1). Although a previous study suggested that two single-nucleotide polymorphisms in STK39 gene may be prognosis factor for overall survival of early-stage NSCLC [10], the expression and biological roles of STK39 in NSCLC have not been clarified. The current study provides insights into the oncogenic role of STK39 in NSCLC through analysis of clinical subjects, and *in vitro* and *in vivo* functional experiments.

The article "Role of high expression levels of STK39 in the growth, migration and invasion of non-small cell type lung cancer cells" was retracted in 2026. Reasons: plagiarized images; duplicated images; overlap with other authors' work; original data or images not available.

Firstly, the clinical data showed that STK39 mRNA was overexpressed in NSCLC tissues that was supported by the expression data from TCGA. Moreover, STK39 protein expression was associated with tumor size, tumor stage, lymph node metastasis and patients' overall survival (Table 1 and Figure 2). Our findings suggested a possible clinical value of STK39 in NSCLC although a more in-depth analysis with more cases was needed. Previous microarray studies [9,14] have identified that lower STK39 mRNA expression was closely related with prostate cancer metastasis, as well as tumor relapse and resistance to certain chemotherapy agents in breast cancer. This discrepancy suggest STK39 may play different role in various malignant tumors.

Further, we explored the biological role of STK39 in NSCLC. Uncontrolled cell proliferation, caused by the aberrant cell cycle progression and resistance to cell apoptosis, is one of the main characteristics of malignancies [15]. Here, knockdown of STK39 in NCI-358 and NCI-H1975 cells suppressed cell growth (Figure 3), inhibited cell cycle progression and induced cell apoptosis (Figure 4). On the contrary, ectopic expression of STK39 in A549 cells caused an inverse effect. Then *in vivo* xenograft tumor formation study (Figure 7) further confirmed our findings of the *in vitro* experiments. CDC25A (a G1/S transition regulator [16, 17]) and PCNA [18] (a proliferation marker) are overexpressed in NSCLC tissues. The prognostic value of Bcl-2 (an anti-apoptosis factor) and Bax (a proapoptotic factor) in NSCLC has also been reported [19, 20]. The expression of the above proteins (Figure 6A) in STK39 knockdown or overexpression cells was consistent with the results of cell cycle and cell apoptosis. These data suggested that STK39 exerted a promotion role on NSCLC cell proliferation via accelerating cell cycle transition and suppressing cell apoptosis. Another characteristic of malignancies is highly metastatic potential [15]. *In vitro* Transwell assays showed that knockdown of STK39 in NCI-358 and NCI-H1975 cells suppressed cell migration and invasion, whereas STK39 overexpression in A549 cells had a promotion effects (Figure 5). MMP-2, MMP-9 [21, 22], snail [23] and E-cadherin [24], important regulators of metastasis, have been found closely related with the prognosis of NSCLC patients. The levels of the above 4 proteins (Figure 6A) in STK39 knockdown or overexpression cells were consistent with the results of Transwell assays. In summary, our data suggest that STK39 plays an oncogenic role in NSCLC progression.

The article "Role of high expression levels of STK39 in the growth, migration and invasion of non-small cell type lung cancer cells" was retracted in 2026. Reasons: plagiarized images; duplicated images; overlap with other authors' work; original data or images not available.

The MAPK pathways play key roles in the regulation of diverse responses, including cell growth, transformation, stress responses and apoptosis. p38 pathway is one of three well-known MAPK pathways [25]. A previous study indicated that p38 is selectively activated in human NSCLC [13]. STK39 can specifically activate the p38 pathway [8]. Here, p38 phosphorylation was inhibited in STK39 knockdown condition, while enhanced in STK39 overexpression cells (Figure 6B). Thus, we speculated that STK39 may exert its biological function through p38 pathways.

In summary, our study suggest that STK39 plays key roles in proliferation, migration and invasion of NSCLC cells, and p38 signal pathway might be involved in the biological function of STK39. STK39 overexpression may serve as an unfavorable progression indicator for NSCLC.

## MATERIALS AND METHODS

### Patients and tissue samples

A total of 135 patients who underwent tumor resection of clinical stage I, II or III NSCLC at Shanghai General Hospital from January 2006 through December 2007 were included in our study. Institutional review board approval and the participants' written informed consent were obtained. The patients had not received chemotherapy or radiation before surgery. Follow-up data and clinical information, such as age, gender, tumor size, tumor type, tumor stage and lymph node metastasis were obtained by review of medical records of the patients. They consisted of 72 males and 63 females and the median age of the participants was 61 years (ranging from 35 to 81 years). The cohort consisted of 71 squamous cell carcinoma (SCC), 46 adenocarcinoma (ADC), and 18 large cell carcinoma (LCC). 40 pairs of fresh NSCLC and matched non-cancerous tissue samples obtained at surgery were immediately frozen and used for RNA sequencing or real-time PCR analysis of STK39 mRNA expression. 135 Paraffin-embedded NSCLC specimens were collected for IHC analysis of STK39 protein expression.

### RNA sequencing

Total RNA was extracted from 10 paired samples using the TRIzol reagent (Invitrogen, Carlsbad, CA, USA) in accordance to the manufacturer's protocol and quantified by ND1000 Spectrophotometer (NanoDrop Technologies, Wilmington, DE). The cDNA libraries were prepared by using mRNA-Seq Sample Prep Kit (Illumina, San Diego, CA, USA). RNA sequencing was performed using Illumina Genome Analyzer using the standard protocol. Sequencing data were converted to FASTQ files using Illumina CASAVA (v.1.8.2) and deposited in NCBI's Sequence Read Archive database (http://www.ncbi.nlm.nih.gov/sra, AC: SRP075725).

The article "Role of high expression levels of STK39 in the growth, migration and invasion of non-small cell type lung cancer cells" was retracted in 2026. Reasons: plagiarized images; duplicated images; overlap with other authors' work; original data or images not available.

### Bioinformatics analysis

Gene set enrichment analysis (GSEA) was performed based on our RNA-seq data by using GSEA version 2.0 from the Broad Institute at MIT as previously described [26]. Gene set permutations were performed 1000 times, and the pathway set list is sorted by the Normalized Enrichment Score (NES).

### Real-time PCR

Total RNA was extracted from 40 paired samples by using TRIzol reagent and treated with DNase I (Roche, Indianapolis, IN, USA) to remove genomic DNA contamination. The extracted RNA (2 μg) was reversely transcribed into cDNA with random primers and cDNA synthesis kit (Thermo Fisher, Rockford, IL, USA). Real-time PCR was done with Maxima SYBR Green qPCR Master Mixes (Thermo Fisher Scientific) on ABI 7300 system (Applied Biosystem, Foster City, CA, USA). GAPDH was used as an internal control. The PCR primers were as follows: STK39 5′- TCTGCTGGCTTGGTGGATG -3′ and 5′- AGGGAGGGTTGAAGGGAGTAG -3′; GAPDH 5′-CACCCACTCCTCCACCTTTG-3′ and 5′- CCACC ACCCTGTTGCTGTAG -3′. STK39 mRNA expression was calculated using the 2^−ΔΔCt^ method.

### IHC staining to assess STK39 protein expression

STK39 protein expression was assessed by IHC staining. Briefly, paraffin-embedded NSCLC specimens were sectioned into 5-μm-thick slices. Sections were then deparaffinized with xylene and rehydrated with a graded series of ethyl alcohol. Antigen retrieval was done by microwave treatment in 0.01 M sodium citrate buffer (pH 6.0) for 10 min. Endogenous peroxidase was inactivated by treatment with 0.3% hydrogen peroxide for 20 min. After incubation with antibody against STK39 (Abcam, Cambridge, MA, USA; 1:50 dilution) for 1 h at room temperature, the slides were then washed in PBS and incubated with horseradish peroxidase (HRP) conjugated secondary antibody for 30 min. After washing in PBS, immunoreactivity was developed by diaminobenzidine tetrahydrochloride (DAB) solution (Vector Laboratories, Burlingame, CA, USA). The tumor specimen was then counterstained with hematoxylin. The staining pattern were categorized into two groups: lower expression group (less than 20% of tumor cells were positively stained) and higher expression group (more than 20% of tumor cells were positively stained).

### Cell culture

Human NSCLC cell lines, NCI-H446, NCI-H358, NCI-H1975, NCI-H292 and A549 were obtained from cell bank of Shanghai Biology Institute, Chinese Academy of Science (Shanghai, China). NCI-H446, NCI-H358, NCI-H292 and NCI-H1975 cells were cultured in RPMI 1640 (Life Technologies, Carlsbad, CA, USA), while A549 cells were cultured in DMEM (Life Technologies). All culture media were supplemented with 10% fetal bovine serum (FBS, Life Technologies), 1% penicillin/streptomycin, and 2 mM L-glutamine (Life Technologies).

The article "Role of high expression levels of STK39 in the growth, migration and invasion of non-small cell type lung cancer cells" was retracted in 2026. Reasons: plagiarized images; duplicated images; overlap with other authors' work; original data or images not available.

### Small interfering RNAs (siRNAs) and lentiviruses

Three siRNAs targeting human STK39 (siRNA1: 5′- GAGGUUCAAUGUUGGAUAU -3′, siRNA2: 5′- CUCCCAUGAAAGUGUUAAU-3′ and siRNA3: 5′- CCCACCCAAUGCUAAUGAA -3′) and a non-specific control siRNA sequence (siNC, 5′-UUCUCCGAACGUGUCACGU-3′) were synthesized by Genepharm Technologies (Shanghai, China), transiently transfected into NCI-H358 and NCI-H1975 cells using Lipofectamine 2000 (Invitrogen, Carlsbad, CA, USA) per the manufacturer's instructions.

The polynucleotide of siRNA3 and siNC was synthesized and inserted into PLKO.1 vector (Addgene, Cambridge, MA, USA). The full-length STK39 were cloned into the expression vector pLVX-puro (Clontech, Palo Alto, CA, USA) by Genewiz Company (Shanghai, China). STK39 knockdown lentivirus (shSTK39), STK39 expressing (STK39) and control (shNC and Vector) lentivirus were generated as described previously [27].

### Western blot analysis

Protein extracts were prepared by using RIPA lysis buffer with freshly added protease inhibitor cocktail (Sigma, St. Louis, MO, USA) [26], separated by SDS-PAGE gel and transferred onto a nitrocellulose membrane (Millipore, Bredford, USA). After blocking with 5% skim milk, the membrane was incubated with primary antibodies [anti-STK39, anti-MMP-2 and anti-MMP-9 (Abcam, Cambridge, MA, USA); anti-PCNA, anti-CDC25A, anti-Snail, anti-E-cadherin, anti-p38, anti-p-p38 and anti-GAPDH (Cell Signaling, Danvers, MA, USA); anti-Bcl-2 and anti-Bax (Santa Cruz Biotech., Santa Cruz, CA, USA)] overnight at 4°C and then incubated with corresponding HRP-conjugated secondary antibody (Beyotime, Shanghai, China) according to the manufacturers' instructions. Signals were detected with enhanced chemiluminescence system (Bio-Rad, Richmond, CA, USA).

### Cell proliferation assay

NCI-H358, NCI-H1975 and A549 cells were seeded in 96-well plates (2 × 10^3^ cells per well). NCI-H358 and NCI-H1975 cells were transfected with siRNA3 or siNC, while A549 were infected with STK39 expressing or Vector lentivirus. After incubation for 0, 24, 48 and 72 h, 10% CCK-8 reagent (Dojindo Lab, Kumamoto, Japan) was added to each well at 37°C for another 1 h. Optical density values (OD) were measured at wavelength 450 nm using a microplate reader (Bio-Rad).

### Evaluation of cell cycle distribution

Cells were harvested at 48 h after siRNA transfection or viral infection. After washing with PBS, the cells were fixed in ice-cold 70% ethanol at −20°C. The fixed cells were washed with PBS and incubated with ribonuclease A (Sigma) and PI (0.05 mg/ml, Sigma) at room temperature for 30 min. DNA content was analyzed on a flow cytometer (BD Biosciences, Franklin Lakes, NJ, USA).

The article "Role of high expression levels of STK39 in the growth, migration and invasion of non-small cell type lung cancer cells" was retracted in 2026. Reasons: plagiarized images; duplicated images; overlap with other authors' work; original data or images not available.

### Analysis of cell apoptosis by flow cytometry

Cells were harvested at 48 h after siRNA transfection or viral infection, washed with PBS, double stained with Annexin V-FITC and PI kit (BD Biosciences), and analyzed on a flow cytometer (BD Biosciences).

### Boyden chamber assay for migration and invasion

Boyden chambers containing 8 μm pore filters (Coring Incorporated, NY, USA) were used for cell migration and invasion assays.

For migration assay, cells cultured on 60-mm diameter dish were treated as described above. After 24 h, cells were serum starved for 24 h, and then 5 × 10^4^ cells in 500 μL serum-free medium were added to the upper chambers, with 500 μL medium containing 10% FBS adding to the lower chambers. After 24 h of incubation, non-migrating cells were completely removed. Migrated cells were fixed in 4% paraformaldehyde, stained with 0.2% crystal violet and counted in five random fields under an Olympus inverted microscope (Lake Success, NY, USA).

Invasion assay was performed as migration assay, except that the upper chamber was pre-coated with 1 mg/ml Matrigel (BD Biosciences).

### Establishment of stable cell lines and tumorigenicity assay

NCI-H358 cells were infected with STK39 knockdown lentivirus (shSTK39) or control lentivirus (shNC). Stable cell lines were obtained by puromycin (Sigma) selection.

The animal study was performed in accordance with the Guidelines for animal experiments of Shanghai Jiao Tong University. BALB/c nude mice aged 4–5 weeks old (Shanghai Laboratory Animal Company, Shanghai, China) were housed in specific- pathogen free conditions under constant humidity and temperature. NCI-H358 cells stably transducted with shSTK39 or shNC were harvested and subcutaneously injected into the right flank of nude mice (2 × 10^6^). Tumor size was monitored every three days by measuring the largest and smallest diameter of the formed tumor. The volume of the tumors was calculated with the following formula: volume = 1/2 × (largest diameter) × (smallest diameter)^2^. 27 days later, the mice were sacrificed and the tumors were recovered. Formalin-fixed, paraffin-embedded tumor sections were stained with anti- Ki67 (Abcam) or analyzed by terminal deoxynucleotidyl transferase–mediated dUTP nick-end labeling (TUNEL, Roche).

### Statistical analysis

All statistical analyses were done with Graphapad Prism software Version 6.0 (San Diego, CA, USA). Student's *t* test was carried out to determine the statistical significance of STK39 expression between different groups. Fisher's exact test was performed to evaluate the relationship between STK39 protein expression and clinicopathological features. Kaplan-Meier survival cures were generated for NSCLC patients with lower or higher STK39 expression, and the difference was analyzed by log-rank test. All *in vitro* experiments were run in triplicates and repeated at least three times. ANOVA test was done to check the statistical significance of *in vitro* cell functional experiments and *in vivo* animal experiments. Statistical significance was set at *P* < 0.05.

The article "Role of high expression levels of STK39 in the growth, migration and invasion of non-small cell type lung cancer cells" was retracted in 2026. Reasons: plagiarized images; duplicated images; overlap with other authors' work; original data or images not available.

## SUPPLEMENTARY MATERIALS FIGURES AND TABLES









## References

[1] Jemal A, Siegel R, Ward E, Hao Y, Xu J, Thun MJ (2009). Cancer statistics, 2009. CA Cancer J Clin.

[2] Jemal A, Bray F, Center MM, Ferlay J, Ward E, Forman D (2011). Global cancer statistics. CA Cancer J Clin.

[3] Koudelakova V, Kneblova M, Trojanec R, Drabek J, Hajduch M (2013). Non-small cell lung cancer—genetic predictors. Biomedical papers of the Medical Faculty of the University Palacky, Olomouc, Czechoslovakia.

[4] Wang Z, Gerstein M, Snyder M (2009). RNA-Seq: a revolutionary tool for transcriptomics. Nature reviews Genetics.

[5] Meyerson M, Gabriel S, Getz G (2010). Advances in understanding cancer genomes through second-generation sequencing. Nature Reviews Genetics.

[6] Mutz K-O, Heilkenbrinker A, Lönne M, Walter J-G, Stahl F (2013). Transcriptome analysis using next-generation sequencing. Current opinion in biotechnology.

[7] Ramoz N, Cai G, Reichert JG, Silverman JM, Buxbaum JD (2008). An analysis of candidate autism loci on chromosome 2q24-q33: evidence for association to the STK39 gene. American journal of medical genetics Part B, Neuropsychiatric genetics.

[8] Johnston AM, Naselli G, Gonez LJ, Martin RM, Harrison LC, DeAizpurua HJ (2000). SPAK, a STE20/SPS1-related kinase that activates the p38 pathway. Oncogene.

[9] Hendriksen PJ, Dits NF, Kokame K, Veldhoven A, van Weerden WM, Bangma CH, Trapman J, Jenster G (2006). Evolution of the androgen receptor pathway during progression of prostate cancer. Cancer research.

[10] Huang YT, Heist RS, Chirieac LR, Lin X, Skaug V, Zienolddiny S, Haugen A, Wu MC, Wang Z, Su L, Asomaning K, Christiani DC (2009). Genome-wide analysis of survival in early-stage non-small-cell lung cancer. Journal of clinical oncology.

[11] Polek TC, Talpaz M, Spivak-Kroizman TR (2006). TRAIL-induced cleavage and inactivation of SPAK sensitizes cells to apoptosis. Biochemical and biophysical research communications.

[12] Balatoni CE, Dawson DW, Suh J, Sherman MH, Sanders G, Hong JS, Frank MJ, Malone CS, Said JW, Teitell MA (2009). Epigenetic silencing of Stk39 in B-cell lymphoma inhibits apoptosis from genotoxic stress. The American journal of pathology.

The article "Role of high expression levels of STK39 in the growth, migration and invasion of non-small cell type lung cancer cells" was retracted in 2026. Reasons: plagiarized images; duplicated images; overlap with other authors' work; original data or images not available.

[13] Greenberg AK, Basu S, Hu J, Yie TA, Tchou-Wong KM, Rom WN, Lee TC (2002). Selective p38 activation in human non-small cell lung cancer. American journal of respiratory cell and molecular biology.

[14] Cleator S, Tsimelzon A, Ashworth A, Dowsett M, Dexter T, Powles T, Hilsenbeck S, Wong H, Osborne CK, O'Connell P, Chang JC (2006). Gene expression patterns for doxorubicin (Adriamycin) and cyclophosphamide (cytoxan) (AC) response and resistance. Breast cancer research and treatment.

[15] Hanahan D, Weinberg RA (2011). Hallmarks of cancer: the next generation. Cell.

[16] Blomberg I, Hoffmann I (1999). Ectopic expression of Cdc25A accelerates the G1/S transition and leads to premature activation of cyclin E-and cyclin A-dependent kinases. Molecular and cellular biology.

[17] Wu W, Fan YH, Kemp BL, Walsh G, Mao L (1998). Overexpression of cdc25A and cdc25B is frequent in primary non-small cell lung cancer but is not associated with overexpression of c-myc. Cancer research.

[18] Nguyen VN, Miřejovský P, Miejovský T, Melínová L, Mandys V (2000). Expression of cyclin D1, Ki-67 and PCNA in non-small cell lung cancer: prognostic significance and comparison with p53 and bcl-2. Acta histochemica.

[19] Apolinario RM, van der Valk P, de Jong JS, Deville W, van Ark-Otte J, Dingemans AM, van Mourik JC, Postmus PE, Pinedo HM, Giaccone G (1997). Prognostic value of the expression of p53, bcl-2, and bax oncoproteins, and neovascularization in patients with radically resected non-small-cell lung cancer. Journal of clinical oncology.

[20] Fontanini G, Vignati S, Bigini D, Mussi A, Lucchi M, Angeletti CA, Basolo F, Bevilacqua G (1995). Bcl-2 protein: a prognostic factor inversely correlated to p53 in non-small-cell lung cancer. British journal of cancer.

[21] Passlick B, Sienel W, Seen-Hibler R, Wockel W, Thetter O, Mutschler W, Pantel K (2000). Overexpression of matrix metalloproteinase 2 predicts unfavorable outcome in early-stage non-small cell lung cancer. Clinical cancer research.

[22] Iniesta P, Moran A, De Juan C, Gomez A, Hernando F, Garcia-Aranda C, Frias C, Diaz-Lopez A, Rodriguez-Jimenez FJ, Balibrea JL, Benito M (2007). Biological and clinical significance of MMP-2, MMP-9, TIMP-1 and TIMP-2 in non-small cell lung cancer. Oncology reports.

[23] Hung JJ, Yang MH, Hsu HS, Hsu WH, Liu JS, Wu KJ (2009). Prognostic significance of hypoxia-inducible factor-1alpha, TWIST1 and Snail expression in resectable non-small cell lung cancer. Thorax.

[24] Sulzer MA, Leers MP, van Noord JA, Bollen EC, Theunissen PH (1998). Reduced E-cadherin expression is associated with increased lymph node metastasis and unfavorable prognosis in non-small cell lung cancer. American journal of respiratory and critical care medicine.

The article "Role of high expression levels of STK39 in the growth, migration and invasion of non-small cell type lung cancer cells" was retracted in 2026. Reasons: plagiarized images; duplicated images; overlap with other authors' work; original data or images not available.

[25] Seger R, Krebs EG (1995). The MAPK signaling cascade. The FASEB journal.

[26] Qiao W, Han Y, Jin W, Tian M, Chen P, Min J, Hu H, Xu B, Zhu W, Xiong L (2015). Overexpression and biological function of TMEM48 in non-small cell lung carcinoma. Tumor Biology.

[27] Moffat J, Grueneberg DA, Yang X, Kim SY, Kloepfer AM, Hinkle G, Piqani B, Eisenhaure TM, Luo B, Grenier JK, Carpenter AE, Foo SY, Stewart SA (2006). A lentiviral RNAi library for human and mouse genes applied to an arrayed viral high-content screen. Cell.

